The article "Bacteriophages Infecting Propionibacterium acnes" was published in 2013. Journal: Biomed Res Int.

# Bacteriophages Infecting *Propionibacterium acnes*

**DOI:** 10.1155/2013/705741

**Published:** 2013-04-11

**Authors:** Holger Brüggemann, Rolf Lood

**Affiliations:** ^1^Department of Biomedicine, Aarhus University, 8000 Aarhus C, Denmark; ^2^Laboratory of Bacterial Pathogenesis and Immunology, The Rockefeller University, 1230 York Avenue, New York, NY 10065, USA

## Abstract

Viruses specifically infecting bacteria, or bacteriophages, are the most common biological entity in the biosphere. As such, they greatly influence bacteria, both in terms of enhancing their virulence and in terms of killing them. Since the first identification of bacteriophages in the beginning of the 20th century, researchers have been fascinated by these microorganisms and their ability to eradicate bacteria. In this review, we will cover the history of the *Propionibacterium acnes* bacteriophage research and point out how bacteriophage research has been an important part of the research on *P. acnes* itself. We will further discuss recent findings from phage genome sequencing and the identification of phage sequence signatures in clustered regularly interspaced short palindromic repeats (CRISPRs). Finally, the potential to use *P. acnes* bacteriophages as a therapeutic strategy to combat *P. acnes*-associated diseases will be discussed.

## 1. Introduction 

Bacteriophages are everywhere! These bacteria-infecting viruses have been isolated in high quantities from many different sources as water [1], soil [2], desert [3], hot springs [4], and humans [5, 6]. They are considered to be the most common biological entity in the biosphere [7], outnumbering bacteria 10 : 1 [8]. Furthermore, phages can be found as prophages inserted into bacterial genomes [9].

Bacteriophages, or phages for short, usually have a narrow host range [10] even though there are reports of phages infecting different species [11, 12]. During infection of a bacterium, a phage has two principal life cycles it can enter—the lytic cycle and the lysogenic cycle (Figure 1). Both cycles are initiated by the attachment of the phage to a surface structure, which usually is species- and even strain-specific [10]. After attachment, the phage will inject its genetic material, which could be either DNA or RNA [13]. After this injection, the phage can enter several different life cycles, with the lytic and lysogenic life cycle being the most common.

While all phages are capable of entering the lytic cycle (virulent phages), some phages (temperate phages) can also enter the lysogenic cycle. The latter requires either the integration of the phage genome into the bacterial host chromosome or, less common, the maintenance of the phage genome as a stable extrachromosomal element [14–16]. Even though several factors have been identified that regulate which cycle is initiated, such as certain phage proteins (e.g., integrases) and environmental factors, this regulatory circuit is still poorly understood [17]. A temperate phage in this state is called a prophage, regardless of whether or not it is integrated; it can be dormant for several bacterial generations [18]. Despite the burden of carrying additional genetic material, bacteria can benefit from prophages, for example, in terms of virulence; a well-known example is the cholera toxin [19] encoded on the CTXphi phage, which can be integrated into the *Vibrio cholera* chromosome. 

The article "Bacteriophages Infecting Propionibacterium acnes" was published in 2013. Journal: Biomed Res Int.

The lytic cycle results in production of phage particles; at the end of the cycle, the lysis cassette of the phage is expressed, producing a holin and a lysine [20], except in the unusual case of filamentous phages that do not lyse their hosts [21, 22]. The holin forms a pore in the inner membrane, enabling the peptidoglycan-degrading lysin to get access to its target; this results in bacterial lysis and eventually in the release of new mature phage progeny. 

Besides these well-established life cycles, other less-defined life cycles exist. One of them is commonly called pseudolysogeny but has also been called “persistent infection” and “carrier-state” [23, 24]; they all describe a similar phenomenon. In the pseudolysogenic cycle, the phage DNA is not integrated but exists as an unstable extrachromosomal plasmid that can be carried by a small bacterial population. The regulation of pseudolysogeny and its effects for the host are still not well understood [23]. Another phage life cycle with relevance for *Propionibacteria* is a chronic infectious state caused by filamentous phages [25]. During this cycle, the phage replicates inside its host, but will not lyse it. Rather, it will form a small pore in the cell wall and continuously release mature phages. Readers with a more general interest in different phage life cycles and genomics of phages are referred to the reviews by Weinbauer [23] and Krupovic et al. [26], respectively.

New bacteriophages of members of the human microbiota have been identified in recent years by means of large-scale sequencing. Interesting examples with potential applications are phages infecting *P. acnes*, a predominant member of the skin microbiota. Even though being considered a skin commensal, *P. acnes* is associated with skin disorders such as acne [27], and potentially with other important diseases, for example, prostate cancer [28, 29]. Due to its ability to form biofilms [30], as well as an increasing resistance to several commonly used antibiotics [31], the potential of using phages to treat this opportunistic pathogen has been raised.

The article "Bacteriophages Infecting Propionibacterium acnes" was published in 2013. Journal: Biomed Res Int.

## 2. *Propionibacterium acnes* Bacteriophages

### 2.1. Identification of *P. acnes* Phages

The first reported phage in the species *Corynebacterium acnes*, a species which largely overlaps with todays' *P. acnes*, was identified already in 1964 by Brzin [35]. In 1968, Zierdt et al. isolated a new *C. acnes* phage, designated 174 [36]. This phage, isolated from the ATCC strain 11827, formed spontaneous plaques on a lawn of *C. acnes* [36]. At that time, the phages were not characterized any further but were used to gain clarity about the classification of the families *Corynebacterium* and *Propionibacterium* [36]. Using phage 174, the authors were able to verify that 88% of the bacteria classified as *C. acnes *indeed were sensitive to the phage, while *Corynebacterium granulosum *and *Corynebacterium lymphophilum* were insensitive to the phage [36]. It should be noted that some of the isolates characterized as *C. acnes* at that time were likely not *P. acnes*, due to differences in characteristics as indole reactions and gelatinase activity. In the years to follow, more researchers used phages to distinguish *C. acnes* from *Corynebacterium avidum *and *C. granulosum* [37–40]. 

Marples and McGinley were able to verify that the morphology of colonies of different corynebacteria correlated with phage sensitivity [41] and thus further stressed that corynebacteria should be further divided into different families. Furthermore, in 1975, Jong et al. used 13 different *P. acnes* phages to divide their collection of propionibacteria into different groups based on their sensitivity to the phages, generating 7 distinct bacterial phage types [42], and also concluded that other propionibacteria (e.g., *Propionibacterium granulosum *and *Propionibacterium avidum*) were resistant to all investigated phages [42]. Other later studies further extended the scheme by adding more phages [43]. Similar typing schemes have also been conducted more recently [33]; however, the value of such studies is questionable since most *P. acnes* strains are sensitive to all phages. In the study by Jong et al., 46 out of 58 strains belonged to the same phage type, even though 13 different phages were tested [42], indicating that the use of phages to (sub-) type *P. acnes* has a limited value. This conclusion was further supported by Voss who noticed that strains susceptible to phage 174 were also prone to be susceptible to phage 26 [40]. Interestingly, it has been noted at that time that certain bacterial phage types were associated with disease, with a higher abundance of specific phage types in inflamed pustules (88%) and acne (73%), as compared to controls (55%) [44]. 

The article "Bacteriophages Infecting Propionibacterium acnes" was published in 2013. Journal: Biomed Res Int.

While the use of phages to divide *P. acnes* into different groups might be outdated, due to current genetic techniques of higher efficiency and sensitivity, such as multilocus sequence typing (MLST) [45, 46], the former is still of importance and has implications for phage therapy, which will be discussed later in this review.

### 2.2. Isolation of *P. acnes* Phages

Bacteriophages can usually be isolated from the same sites as their hosts, since they depend on their hosts for replication. Thus, *P. acnes* phages can be isolated from lipid rich areas of human skin, mainly the forehead and nostrils [47, 48], where they can reach concentrations of up to 10^7^ plaque forming units (pfu) from a swab from the nostrils [48]. Furthermore, Marples et al. concluded that females carried fewer *P. acnes* phages than men, which also correlated with the lower abundance of *P. acnes* on females [48]. Besides being able to isolate *P. acnes* phages from general parts of the skin, comedones harbor a high concentration of *P. acnes* specific phages, with detectable phages in 26%–30% of the investigated samples [39, 49]. Using next generation sequencing, Sharon et al. were able to demonstrate the presence of *Propionibacterium* phages in the gastrointestinal tract using a metagenomics approach [50]. A similar approach also allowed Willner et al. to specifically identify *P. acnes* phages in the oral cavity [51].

### 2.3. Morphology of *P. acnes* Phages

The first micrographs of phages infecting *P. acnes* were published in 1974 by Marples [47] and Zierdt [52]. While they both identified phages with a morphology similar to Siphoviruses, Zierdt identified only smaller phages with isometric heads (42–44 nm) and 130 nm long tails [52] while Marples also identified phages with considerably larger heads (67 nm); these phages were associated with different plaque morphologies [47]. In 1978, Webster and Cummins confirmed that phages with 72 nm heads and long tails (196 × 10 nm) existed [53]. Furthermore, Webster and Cummins showed that phages with even larger heads (90 nm in diameter) were present in their collection, with a shorter and wider tail (175 × 15 nm) [53]. Even though the general morphology is identical, later studies have only been able to identify phages with head sizes of around 50–55 nm in diameter, and with a tail of 150 × 10 nm (Figure 2) [33, 54, 55]. However, it is currently not known if the differences in observed phage morphologies are due to technical reasons (e.g., morphological changes due to differences in sample preparations for electron microscopy), or if they truly represent extinct or not yet reisolated phages.

The article "Bacteriophages Infecting Propionibacterium acnes" was published in 2013. Journal: Biomed Res Int.

### 2.4. Phages Infecting Other Propionibacteria

Besides the study of phages infecting *P. acnes*, phages infecting other propionibacteria have also gained some interest, mainly due to their importance in the dairy industry. Gautier et al. showed in two different studies in 1995 that phages infecting *Propionibacterium freudenreichii* were present in more than 50% of samples from different cheeses [56, 57]. The phages were similar in morphology to those infecting *P. acnes*, for example, identical to Siphoviruses. One-step growth curves suggested a latent period of 6-7 hours with a burst size of 60 phages per bacterium [57], which is considerably slower than that reported for a *P. acnes* phage, with a latent period of only 1 hour, even though the burst size is slightly lower [52]. 

There exist several differences between the two groups; while integrated inducible prophages in *P. acnes* still remain to be identified, active prophages have been detected in several dairy Propionibacteria (e.g., *P. freudenreichii* subsp. *freudenreichii*, *P. freudenreichii* subsp. *shermanii*, *Propionibacterium jensenii,* and *Propionibacterium thoenii*); Southern blot-based detection and induction by either mitomycin C or UV were used to confirm their presence and functionality [58]. Furthermore, phages infecting *P. acnes* have all been classified as dsDNA carrying siphoviruses; in contrast, *P. freudenreichii* can also be infected by ssDNA filamentous phages [25]. These are 620 × 12 nm in size and have a small genome of 5,806 bp encoding 10 putative genes with similarities to genes of Gram-negative filamentous phages [25].

### 2.5. Genomic Analysis of Phages Infecting *P. acnes*

The first sequenced *P. acnes* phage was phage PA6, reported by Farrar et al. in 2007 [54]. Since then, 13 additional phages have been sequenced [34, 55]. They all have a similar genome arrangement (Figure 3), and similar genome lengths ranging from 29,017 to 29,739 bp, with 45–47 encoded putative proteins [55]. The first part of the genome encodes proteins mainly involved in DNA packaging (terminases) and structural proteins; several of the proteins have been experimentally verified to be produced by matrix-assisted laser desorption/ionization time-of-flight (MALDI-TOF) mass spectrometry [34]. This part of the genome is followed by a lysis cassette, encoding a holin and an amidase for the degradation of bacterial peptidoglycan. All these genes are transcribed from the plus strand, while most of the remaining genes, mainly of unknown functions, are transcribed from the minus strand [34, 55]; the latter genes might be involved in DNA regulatory processes [34, 55].

The article "Bacteriophages Infecting Propionibacterium acnes" was published in 2013. Journal: Biomed Res Int.

As was suggested by us, and further emphasized by Marinelli et al., phages infecting *P. acnes* seem to represent a unique, almost clonal lineage of phages with low similarity to other phages [34, 55]. There is an astonishing conservation of different *P. acnes *phage genomes, with a nucleotide identity higher than 85%, despite their isolation from different countries (England, Sweden, and USA) and different times of isolation covering a time span of more than 30 years. It has been speculated that one reason for this conservation might be the specific niche of *P. acnes*, which reduces lateral gene transfer or recombination events [55].

Recently, a phage able to infect the Gram-negative bacterium *Fusobacterium nucleatum* was isolated and partly characterized [59]. A small 500 bp DNA fragment was sequenced and showed more than 90% nucleotide sequence identity to two structural protein-encoding genes of *P. acnes* phages (gp3 and gp4). This finding is striking since *F. nucleatum* belongs to the low-GC bacteria, with a GC content of around 28%, which is in sharp contrast to the high GC bacterium *P. acnes* (60%) and *P. acnes *phages (54%) [55]. Thus, since the GC-content at least in that specific region is vastly different from its *F. nucleatum* host, it might be that the uptake of this phage in *F. nucleatum* represents an evolutionary new event. However, due to the high presence of *P. acnes* phage DNA in the oral cavity [51], it might be that this sequence only represents a contaminating DNA fragment that originates from a *P. acnes* phage, rather than being an actual part of a *F. nucleatum* phage.

### 2.6. Life Cycles of *P. acnes* Phages

The life cycles of the characterized *P. acnes* phages are still not well understood. During the 1970s, several studies tried to characterize the life cycles of phages infecting *P. acnes* but with contradictory results. Pulverer et al. showed in 1973 that 3 out of 63 *P. acnes* strains exhibited spontaneous lysogeny, since they could release infectious phages by spontaneous induction [60]. The addition of the phage-inducing substance mitomycin C released phages from more than 38% of all investigated strains, while UV-induction did not work [60], suggesting true lysogeny. Webster and Cummins came to the same conclusion five years later, even though mitomycin C treatment released phages in only 17% of the strains [53]. Recently, similar studies demonstrated that more than 70% of *P. acnes* could be induced with mitomycin C to generate infectious phages [33]. In contrast, Zierdt could not detect any spontaneously released phages in a large collection of *P. acnes *strains, neither could he show phage induction using mitomycin C [52]. Jong et al. concluded that their data “*from phagetyping were inconclusive, and most of the phage-stocks later proved to be mixtures of virulent and temperate phages*” [42].

The article "Bacteriophages Infecting Propionibacterium acnes" was published in 2013. Journal: Biomed Res Int.

In more recent years, some light has been shed on this question, even though the life cycle of these phages is far from being well understood. From the first phage genome sequence, it could be concluded that the phage PA6 lacked any integrase and repressor and was thus classified as a lytic phage [54]. Still, the phage did generate turbid plaques, sometimes indicative of lysogeny. The same phenomenon was visualized already in 1974 by Zierdt, who concluded that the turbid *P. acnes* colonies within the plaques were still sensitive to the phage, indicating that the bacteria did not acquire any superinfection immunity or general resistance to the phages [52]. Further studies and sequencing of more phage genomes supported the idea that *P. acnes* phages lacked any common lysogenic module [33, 34, 55]. Thus, it was suggested that the phages can be carried for a few generations by the bacterial host in an unstable pseudolysogenic state, without the integration of their genome [34]. 

## 3. Cutaneous Microenvironment and Its Impact on *P. acnes* and Phage Evolution 

Phage genome sequencing revealed a high conservation among *P. acnes*-infecting phages. This corresponds to the low diversity within the *P. acnes* population; type I strains of *P. acnes*, which represent the vast majority on human face and back, show high conservation as judged from their genome sequences [61]. This conservation might be explained by the specialized nice of *P. acnes*. Species diversification is often increased by competition and changing environmental conditions. Such driving forces of evolution are lacking in sebaceous follicles; it has been found that only very few organisms can colonize this lipid-rich niche. In fact, *P. acnes* is often the sole resident in sebaceous follicles [62]. 

Reasons for the prevalence of *P. acnes* are several environmental and physiological parameters that restrict growth in sebaceous follicles, such as local humidity, nutrient availability and accessibility, pH, and temperature. In addition, host defense mechanisms exist, including antimicrobial peptides, proteases, cytokines, and chemokines that can either directly inhibit microbial growth or serve as activators and mediators of the innate and adaptive immune responses. *P. acnes* has adapted to this environment and evolved strategies to survive in such a niche; such strategies include (among others) a strong lipolytic activity, pH regulatory mechanisms [61], biofilm formation [30], and possibly the activation of a dormant state and the escape into host cells [29]. The adaptation and specialization likely resulted in low bacterial diversity, which might be mirrored in a low diversity of *P. acnes*-infecting phages.

The article "Bacteriophages Infecting Propionibacterium acnes" was published in 2013. Journal: Biomed Res Int.

## 4. Cryptic Prophage-Like Genomic Island

None of the currently characterized phages seem to be able to integrate into the *P. acnes* genome. However, genomic data suggests that ancient phages have been able to do so, since several genomes of* P. acnes *(such as strains KPA1701212, 6609, and HL030PA1) harbor a 32 kb genomic region that encodes prophage-related proteins, including proteins similar to a phage-related DNA polymerase and a prophage antirepressor. The 3′-end of this island, encoding a restriction-modification system, might have a different, phage-unrelated origin [63, 64] (Figure 4). The cryptic prophage-like region does not encode proteins with similarity to structural phage proteins, integrases or lysis cassettes [64]. Furthermore, the protein sequences do not exhibit similarity to proteins encoded by functional *P. acnes* phages [34]. Thus, it is likely that these regions represent extinct phage remnants that are not functional anymore.

Most of the prophage-like region-positive strains belong to a specific subtype of *P. acnes* (CC36, type I-2 according to the typing scheme of Lomholt and Kilian, 2010 [27]). Other *P. acnes* strains such as HL025PA1 (type Ia) possess a similar region with a small deletion within a gene encoding a putative DNA methylase that is part of a restriction-modification system at the 3′-end. The 5′-end of the prophage-like region in *P. acnes* also displays high similarity to a putative cryptic prophage region in *P. avidum* ATCC 25577 (Figure 4).

Apart from these putative cryptic prophages, no phages have been reported to be able to integrate in the genome of *P. acnes*. The lack of integration may partly be attributed to the several defense mechanisms that *P. acnes* possess against foreign DNA, among other clustered regularly interspaced short palindromic repeats (CRISPRs).

## 5. *P. acnes* CRISPRs

CRISPRs together with CRISPR-associated (Cas) proteins are an “adaptive immune system” of bacteria and archaea, which can protect the carrier organism from an attack of foreign DNA as part of mobile genetic elements, including phages and plasmids. A prerequisite to a successful defense is the “acquired immunity,” that is, the existence of a CRISPR spacer sequence that originated from the “infecting” mobile genetic element. 

A *cas* gene cluster has been identified in *P. acnes*; it comprises eight genes [65]. These are usually restricted to genomes of type II *P. acnes* strains. Remnants of the *cas* gene cluster can be found in type III strains and even smaller parts (typically a fragment of *cas*1 and *cas*2) in type I strains, indicative of reductive evolution.

The article "Bacteriophages Infecting Propionibacterium acnes" was published in 2013. Journal: Biomed Res Int.

CRISPR spacers of *P. acnes* have been sequenced in type II strains. Our analyses, combined with the study of Marinelli et al. [55] and Fitz-Gibbon et al. [66], revealed 133 spacers in 34 different strains (Supplementary Table 1). Among these 133 spacers, 52 phage-specific spacers were found, representing 16 different sequences of phage genomes (Supplementary Table 2) [55, 65]. These spacers are derived from 12 phage genes and one noncoding region (Figure 3). Interestingly, one spacer sequence is conserved in 14 different phage genomes (Supplementary Table 2) and 17 CRISPR spacers originated from one phage gene (gp16). A similar phenomenon was also reported most recently for *Streptococcus thermophilus *with a strong bias for certain spacers [67]. This is in stark contrast to earlier studies on *Streptococcus*, where no such preferences could be found [68–70]. Thus, there seems to be a bias in some species, where certain phage regions are preferentially processed to be used as CRISPR spacers.

Since only type II strains of *P. acnes* possess CRISPR/*cas* loci, it can be speculated that type I strains should be more sensitive to phage infections. Indeed, already in 1978, Webster and Cummins noticed that type I strains were more susceptible to phage infections [53], which also was demonstrated more recently [33]. Moreover, Marinelli et al. demonstrated that *P. acnes* isolates with spacers similar to phage sequences were significantly more resistant to phage infections, as compared to isolates without phage specific spacers [55]. Thus, this strongly suggests that the phage specific spacers found in *P. acnes* may confer phage resistance. However, the CRISPR system is only one of several defense mechanisms against phage infections that bacteria have developed, and the actual importance of this system for *P. acnes* phage resistance has not been investigated thoroughly yet. 

## 6. *P. acnes* Phage Therapy

Since the discovery of bacteriophages, scientists have been fascinated by their potential as a novel strategy to treat infectious diseases. d'Hérelle investigated this potential already in 1912, and still a century later, the same therapeutic option continues to interest researchers. Still, only a few countries have so far accepted the usage of phages as a therapeutic option in humans, with the phage therapy center in Tblisi, Georgia, being one of the more established places offering phages to treat several infectious diseases [71]. However, the availability of highly efficient antibiotics, a poor understanding of general aspects of phage life cycles, bacterial resistance to phage infection, and a fear that temperate phages might be able to integrate into the human genome and thus contribute to cancer [72] have slowed down the progress in the research field of phage therapy. Besides the possibility that antibodies might clear circulating phages, it has been suggested that phages might be able to bind to human cells, even though this has not been firmly demonstrated yet [73]. More specifically, it has been suggested that phages have a tendency to bind to *β*3 integrins mainly on neoplastic cells, since the addition of anti-*β*3 integrin antibodies inhibited this interaction [74]. These host cell interactions could be mediated via proteins containing Arg-Gly-Asp- (RGD-) like recognition motifs, which are present in the major structural proteins of phages [73]. RGD-containing proteins are known to be able to bind to integrins [75], a strategy employed by certain viruses to gain entrance into human cells [75]. Of interest, two of the major structural proteins of *P. acnes* phages have such domains (gp11 and gp15; major tail and minor tail subunits, resp.). It is currently not known if these phage proteins can indeed bind to human host cell receptors. 

The article "Bacteriophages Infecting Propionibacterium acnes" was published in 2013. Journal: Biomed Res Int.

Another drawback in the field of phage therapy is the fast generation of phage-resistant bacteria. In order to be infectious, the phage needs to attach to the surface (Figure 5), and it is usually this receptor that is mutated in phage-resistant bacteria [76]. In 1973, Pulverer et al. realized that while the main part of a *P. acnes *population was sensitive to phages, a small subpopulation exhibited resistance to all phages [60]. Two years later, Jong et al. came to the same conclusion, demonstrating that around 1.7% of all investigated strains were completely resistant to all phages [42]. However, other studies suggested a much higher resistance rate of up to 15.6% [53] and stressed the possibility that sensitive strains may rapidly develop resistance [36]. 

To evaluate if phage therapy could be successfully applied to clear *P. acnes* from skin sites, a few considerations are needed. In a recent study, Vieira et al. used phages to reduce the colonization of *Pseudomonas aeruginosa ex vivo* on skin with some success. After four hours of treatment, they could see a four-log reduction of *P. aeruginosa*, while the phage concentration had increased, indicating that the phages had been able to replicate on the skin [77]. Even though promising, this *P. aeruginosa* skin infection model does not resemble the actual niche of *P. acnes,* the sebaceous follicles [78]; thus, it might be more difficult for phages to gain access to *P. acnes in vivo*. 

The article "Bacteriophages Infecting Propionibacterium acnes" was published in 2013. Journal: Biomed Res Int.

Besides being implicated in skin diseases, *P. acnes* has also been associated with several clinical conditions due to its biofilm forming ability, mainly on catheters and other orthopaedic materials [79]. In biofilms, *P. acnes* are generally quite resistant to antibiotics and other antibacterial agents [80], and thus it is of importance to investigate if they also are protected against phages. In a 2012 study, Alemayehu et al. found that biofilms formed by *P. aeruginosa* could efficiently be degraded *in vitro *by a cocktail of *P. aeruginosa *specific phages. More importantly, the phages were able to significantly reduce the colonization of *P. aeruginosa *in murine lungs [81], again stressing that phage therapy might prove successful. Furthermore, actual pretreatment of catheters with bacteriophages might further reduce biofilm formation, as was shown in a *Staphylococcus epidermidis* model [82], which might be of therapeutic interest since this bacterium usually can be identified from similar infections as *P. acnes *[83, 84]. 

Even though these *P. aeruginosa *and *S. epidermidis *models show great potential of phage-based therapeutical strategies, the actual biology of *P. acnes *and its phages might complicate such therapies for *P. acnes *infections. In phage therapy, it is of importance to use exclusively lytic phages. However, there is still a lack of understanding on the actual life cycles of *P. acnes* phages; a pseudolysogenic cycle has been suggested to exist [34]. Furthermore, *P. acnes* might easily develop resistance to phages; when they do, they are usually resistant to most, if not all, phages [33, 53]. 

Another problem of *P. acnes* phage therapy might be the unusually high homogeneity seen between different *P. acnes *phages [34, 55]. This homogeneity has been suggested to be due to undefined evolutionary constraint that limits this diversity and thus maintains a phage with little genetic diversity [55]. Initially, this homogeneity might be beneficial, since most isolated phages have a broad activity versus almost all *P. acnes *strains [33], thereby avoiding the necessity of phage typing. However, due to the highly conserved genomes, CRISPR spacers or mutations in the phage host receptor will affect most phages and thus render *P. acnes* resistant to most phages. Usually, when using phage therapy, it is strongly recommended to use phages that bind different receptors (e.g., using a phage cocktail), to lower the risk of developing resistance [85]. Thus, the high homogeneity of the currently isolated phages might limit the efficiency of phage therapy. 

The article "Bacteriophages Infecting Propionibacterium acnes" was published in 2013. Journal: Biomed Res Int.

Finally, for a phage therapy to be successful, many other parameters are of importance, including but not limited to delivery route, time point of delivery, dose, stability of phages, and infection rate *in vivo*. These are parameters that need to be empirically tested. For a more general view of how these factors might influence the success of phage therapy, the reader is referred to a review on this topic by Ryan et al. [86], also suggesting novel methods of how to deliver bacteriophages [87]. For those with a more general interest in phage therapy, the reader is referred to the reviews by Loc-Carrillo and Abedon [88] and Abedon et al. [89]. 

## 7. Conclusions

Much has happened since Twort and d'Hérelle first identified bacteriophages and since Brzin identified the first *P. acnes* phage in 1964. Several more phages have been isolated and visualized in great detail using electron microscopy and have been characterized to some extent. Recently, the genomic era has enabled us to generate a vast amount of sequence data of phages and their bacterial hosts. This already revealed the uniqueness and homogeneity of *P. acnes* phages. However, regardless of the generated data, much is still unknown, in particular when it comes to the interaction between the phage and *P. acnes*. Further studies of these interactions, including the contribution of prophages to bacterial pathogenicity, the life cycles of the phages, and the role of CRISPRs, may eventually allow us to investigate the potential of using phages, or phage-derived molecules, as a therapy against *P. acnes*-associated diseases.

## Supplementary Material

Supplementary Table 1. Identified CRISPR spacers in CRISPR/cas regions of sequenced *P. acnes* strains. Identified spacers from all currently publicly available *P. acnes* genomes were extracted (reference 55, 64, 66) and were screened for homology to known nucleotide sequences.
Supplementary Table 2. Identified CRISPR spacers originating from *P. acnes* phages. Based on all the available CRISPR spacers of *P. acnes* (reference 55, 64, 66, see Supplementary Table 1), spacers with similarities to published *P. acnes* phage genomes were analyzed based on their length, GC content, orientation and localization.

## Figures and Tables

**Figure 1:** Phage life cycles. After attachment, the phage injects all its genetic material through the cell wall into the cytoplasm. The phage might then enter the lytic cycle, where it replicates, produces new mature progeny, and eventually lyses the bacterial cell by the insertion of the pore forming holin in the inner membrane, thus allowing the endolysin to gain access to and degrade peptidoglycan. Certain phages, termed temperate phages, can under the right environmental circumstances instead enter the lysogenic life cycle and either integrate their genetic material into the host chromosome by the use of integrases or exist as stable extrachromosomal plasmids. These phages, so called prophages, are then replicated along with the bacterial chromosome. Once prophages are induced (activated), they will enter the lytic cycle, start to propagate, and eventually lyse their host. The figure is adapted from [32].

The article "Bacteriophages Infecting Propionibacterium acnes" was published in 2013. Journal: Biomed Res Int.

**Figure 2:** Morphology of *P. acnes* phages. All isolated bacteriophages infecting *P. acnes* have been classified as Siphoviruses, due to their long noncontractile tail, and icosahedral heads (a). They also have a base plate with visible tail fibers (b), adhering to certain host receptors. The figure is adapted from [33].

**Figure 3:** Genomic organization of *P. acnes *phages and the location of CRISPR protospacers. All currently sequenced *P. acnes* phage genomes have a length ranging from 29,017 to 29,739 bp. Most of the dsDNA is coding sequence; 45–47 open reading frames (ORFs) exist. In addition, a 1.4 kb noncoding region (27431–28877 in phage PA6) seems to have a regulatory function. Open reading frames (arrows) in gray represent genes for which CRISPR spacers have been identified. The number in the ORFs denotes the actual number of protospacers identified for each gene. For a more specific map, the reader is referred to the Supplementary Table 2. The figure is adapted from [34].

**Figure 4:** Comparison of the prophage-like region in strains of *P. acnes *and* P. avidum*. A few type I-2 and a few type Ia strains like KPA171202 (KPA) and HL025PA1, respectively, possess a prophage-like region, while most type Ia (like strain 266) and type II and type III strains do not contain such a region. *P. avidum* strain ATCC25577 harbors a similar region, though the 3′-end differs in *P. acnes*. The comparison was done using the Artemis Comparison tool (ACT, Sanger Institute).

**Figure 5:** *P. acnes* phage life cycle. The phage first attaches to a receptor present on the surface of the bacterium. Once attached, the phage injects its DNA. The two leftmost phages still have their DNA packed in their head, as visualized as small strands, while the third, rightmost, phage has injected its DNA, and thus the head is deformed during the preparation for electron microscopy. The phage replicates inside its host and eventually produces a holin and a lysin to cause lysis of the bacterium and thus the release of all its content, including mature bacteriophages ready to infect new bacteria. The figure is adapted from [32].
